# Patterns and Predictors of Timely Presentation and Outcomes of Polytrauma Patients Referred to the Emergency Department of a Tertiary Hospital in Tanzania

**DOI:** 10.1155/2022/9611602

**Published:** 2022-11-04

**Authors:** Elishah N. Premji, Said S. Kilindimo, Hendry R. Sawe, Amne O. Yussuf, Alphonce N. Simbila, Hussein K. Manji, Juma A. Mfinanga, Ellen J. Weber

**Affiliations:** ^1^Emergency Medicine Department, Muhimbili University of Health and Allied Science, Dar es Salaam, Tanzania; ^2^Emergency Medicine Department, Muhimbili National Hospital, Dar es Salaam, Tanzania; ^3^Department of Emergency Medicine, University of California, San Francisco, CA, USA

## Abstract

**Background:**

Polytrauma patients require special facilities to care for their injuries. In HICs, these patients are rapidly transferred from the scene or the first-health facility directly to a trauma center. However, in many LMICs, prehospital systems do not exist and there are long delays between arrivals at the first-health facility and the trauma center. We aimed to quantify the delay and determine the predictors of mortality among polytrauma patients. *Methodology*. We consecutively enrolled adult polytrauma patients (≥18 years) with ISS >15 referred to the Emergency Medicine Department of Muhimbili National Hospital, a major trauma center in Tanzania between August 2019 and January 2020. Based on a pilot study, the arrival of >6 hours after injury was considered a delay. The outcome of interest was factors associated with delayed presentation and the association of timeliness with 7-day mortality.

**Results:**

We enrolled 120 (4.5%) referred polytrauma adult patients. The median age was 30 years (IQR 25–39) and the ISS was 29 (IQR 24–34). The majority (85%) were males. While the median time from injury to first-health facility was 40 minutes (IQR 33–50), the median time from injury to arrival at EMD-MNH, was 377 minutes (IQR 314–469). Delayed presentation was noted in more than half (54.2%) of participants, with the odds of dying being 1.4 times higher in the delayed group (95% CI 0.3–5.6). Having a GCS <8 (AOR 16.3 (95% CI 3.1–86.3), hypoxia <92% (AOR 8.3 (95% CI 1.4–50.9), and hypotension <90 mmHg (R 7.3 (95% CI 1.6–33.6) were all independent predictors of mortality.

**Conclusion:**

The majority of polytrauma patients arrive at the tertiary facilities delayed for more than 6 hours and a distance of more than 8 km between facilities is associated with delay. Hypotension, hypoxia, and GCS of less than 8 are independent predictors of poor outcome. In the interim, there is a need to expedite the transfer of polytrauma patients to trauma care capable centers.

## 1. Introduction

Worldwide, trauma contributes significantly to the burden of disease and mortality. According to WHO, 5.8 million trauma victims die from injuries every year and 90% of trauma-related deaths occur in LMICs [1]. In sub-Saharan Africa, mortality due to polytrauma ranges from 5.5% to 33% [2, 3].

A primary concept in the trauma literature is the “golden hour.” This is the initial 60 minutes from the time of injury of a trauma patient to definitive care, during which physicians have the greatest chance of reversing the life-threatening effects of trauma. This concept may not be feasible in LMICs which suffer from long distances between scenes of injury and hospitals; poor road infrastructure; lack of prehospital emergency medical services (EMS); and lack of trauma centers [4].

Most preventable deaths due to multiple traumas are attributed either to a delay in arrival at a primary care facility or a timely referral to a specialized center [5]. Research in both LMICs and HICs has shown that delay is more frequent in trauma victims presenting during the night at peripheral facilities [2], having higher injury severity scores [6], and having sustained injury in a public place [7].

Tanzania lacks a formal prehospital trauma system, which is important in the initial care of acutely injured patients [8]. If severely injured patients are initially transported to a hospital not properly equipped to care for them, the initial stabilization needs to be performed quickly and plans should be made for prompt transfer to a trauma center [9]. A study conducted in Tanzania by Lucumay et al. revealed gaps in capability for caring of these trauma patients in most first-health facilities [10], suggesting urgent transfer to a hospital that has the proper skills and resources for care is the ideal practice in LMIC.

Several factors may aid in the rapid transfer of patients but may also serve as independent factors of the severity of injuries, and in turn, influence the outcome of trauma patients. A low GCS [11–13], high ISS [14–16], and derangement in vital signs (hypotension and hypoxia) are some major factors [11, 17].

We aimed to quantify the delay, determinants, associated factors, and predictors of poor outcome among polytrauma patients presenting to EMD-MNH.

## 2. Methods

### 2.1. Study Design

This was a prospective cohort study of referred adult polytrauma patients conducted at EMD-MNH between August 2019 and January 2020.

### 2.2. Study Setting

The study was conducted at EMD-MNH, which is a public, tertiary referral hospital located in Dar es Salaam, Tanzania, with a 1500 bed capacity. The EMD provides emergency care and resuscitation, serving an average of 200 patients a day. About 25% of the received patients are trauma cases. After a standardized approach to trauma patients is carried out, patients are either disposed to a specialized trauma center at MOI within the Muhimbili campus. MOI is a full-capacity center for orthopedic and neurosurgical services within the country. Those with soft tissue (abdominal/chest visceral) as well as facial injuries are cared for by general and maxillofacial surgeries, respectively.

### 2.3. Study Participants

All consenting adult patients, 18 years and older, who had been referred from another health facility with polytrauma, were included. We excluded patients with ISS ≤15, those who presented directly from the scene of injury, patients brought dead on arrival and referrals beyond 24 hours from the time of injury.

### 2.4. Study Protocol

Research assistants were scheduled to collect data on consecutive patients for 24 hours on alternate days. Using referral notes, interviews with patients and/or relatives and the electronic medical record (Wellsoft™) data were collected and recorded on a structured case report form. Participants' information included demographics, referring hospital, mechanism of injury, pattern of injury, time of injury, vital signs, and initial primary survey, and whether any critical interventions were undertaken within 15 minutes of the arrival of the patients were collected. Using the WHO trauma checklist, patients who should have had interventions for stabilization prior to transfer were noted. Also, timings of interest (time of injury, time to arrival at first facility, time from first facility, and time to arrival at EMD) were obtained. To determine their outcome, patients were followed up in a hospital ward or through mobile phone calls if discharged in less than 7 days from the EMD presentation.

### 2.5. Outcomes

The primary outcome was predictors of delay, and the secondary outcomes were associated with delay and 7-day mortality. A pilot study was used to estimate sample size using a 2-proportion dichotomous outcome (delay vs. no delay). 70% of patients were delayed, hence providing a minimum sample size of 108 to estimate effect size.

### 2.6. Data Analysis

Data from the case report form were entered into REDCap (version 7.2.2, Vanderbilt, Nashville, TN, USA) and transferred into the Statistical Package for Social Science (version 25.0, IBM, LTD, North Carolina, USA). Relevant frequencies and tables were generated for categorical variables such as demographics, mechanism and pattern of injury, primary survey, vital signs, and pre-referral stabilization provided. Medians/interquartile ranges were calculated for continuous variables such as distance between facilities, time from injury to arrival at the first hospital, and transfer to MNH. A Pearson chi-square and relative risks were computed for associations between categorical variables and timeliness of presentation. For the secondary outcome, a univariate logistic regression was performed to identify variables associated with 7-day mortality, after which a multivariate logistic regression was completed on variables with a *P* value ≤0.20 in the univariate analysis to highlight independent predictors. A Mann–Whitney *U* test was conducted for timeliness as a continuous variable to assess its effect on 7-day mortality.

## 3. Results

During the study period, a total of 2650 adult trauma patients were attended at the EMD. Among these, 1060 (40%) were triaged as ESI level 1 and 2, of whom 120 patients met the inclusion criteria and were subsequently enrolled. The proportion of referral polytrauma patients was 4.5% and the overall 7-day mortality was 24 (20%) (Figure 1).

### 3.1. Clinical Profile of Referral Polytrauma Patients Who Presented to the EMD-MNH

Among the 120 referral patients with polytrauma, the majority were middle-aged males. The median ISS was 29 (IQR 24–34). The predominant mechanism of injury was a motor vehicle accident, with the motorcycle driver as the most common victim. The frequent pattern of injury was head/neck, followed by long bones/pelvis. Most injuries occur between 8 pm and 8 am. A GCS of 8 or less was seen in a third of the patients. Unstable vital signs were noted as follows: hypoxia (40%), abnormal heart rate (65%) and hypotension (21%). In the primary survey, approximately a third of patients had compromised airways and nearly half had compromised breathing. Over half of the patients required a critical intervention within 15 minutes of arrival at the EMD. Among the prereferral care instituted, none of the 17 patients requiring a chest tube received it at the initial facility. 4 out of 10 patients lacked a cervical spine collar. Endotracheal intubation was performed in only 3 of 41 patients who had indications for this intervention (Table 1).

### 3.2. Referral Characteristics and Timing of Presentation of Referral Polytrauma Patients Presenting to the EMD-MNH, Dar es Salaam, Tanzania

The median distance between facilities was 8.1 km and over half of the patients were referred from regional hospitals. The median time from injury to first hospital was 40 minutes, and the majority arrived at a health facility within the golden hour. The median time from injury to MNH was 6.3 hours (Table 2).

### 3.3. Factors Associated with Timely Presentation of Referral Polytrauma Patients Who Presented to the EMD-MNH, Dar es Salaam, Tanzania

Timely presentation (less than 6 hours post injury) was noted among 55 (45.8%) of patients. The only factor associated with timely presentation was distance, which was less than 8 km between facilities. There was no difference between the timely and late groups with regard to age groups, GCS, ISS, time of injury, location of injury, or need for immediate intervention at MNH-EMD (Table 3).

### 3.4. Predictors of Mortality among Referral Polytrauma Patients Who Presented to the Emergency Department of Muhimbili National Hospital, Dar es Salaam, Tanzania

With univariate and multivariate regression analyses, we found GCS of ≤8, hypoxia of ≤92%, and hypotension of ≤90 mmHg to be independent predictors of mortality among polytrauma patients. However, a delay of more than 6 hours was not a statistically significant predictor of mortality (Table 4).

## 4. Discussion

Using a 6 hour cutoff time from injury to EMD arrival, more than half of patients were delayed (arrived beyond 6 hours), with no statistically significant odds of mortality in those patients who were delayed. Referred polytrauma patients were 4.5% of our total trauma volume seen during the study period, which was not similar to a national study conducted by Sawe et al. on district and regional hospitals which found the prevalence at 5.5% [3]. One possible explanation could be that since our study was conducted at a tertiary level facility, some patients do not make it all the way along the referral system, i.e., die before reaching the tertiary level facilities. In contrast, a study conducted in South Africa found the prevalence of polytrauma to be sixfold higher [2]. A reason for this difference could be the existence of pre-hospital EMS in South Africa to treat and transport acutely sick or injured patients to the hospital as opposed to our setup, which lacks this formal system [2, 18].

The majority of patients arrived at the initial facility during the “golden hour”, yet the median time to reach the EMD, which is a trauma center, was slightly over 6 hours. In contrast, studies conducted in Australia and California have shown that the majority of transferred patients arrive to the major trauma center within 4.5 hours of injury [14, 19, 20]. One would think the delay in transfer might be due to measures needed to stabilize patients at the initial hospital. However, over half of the transferred patients had not received adequate prereferral stabilization and required a critical intervention upon arrival at EMD. Harrington and colleagues in the USA [6] found that only 8% of transferred patients required a critical intervention on arrival to the trauma center.

Endotracheal intubation and chest tubes were not performed in almost all of the patients who required these interventions. Similar results were also observed in a study conducted in South Africa [2], whereby less than 20% of patients received any of these interventions. Several studies conducted in India have confirmed suboptimal levels of prereferral care, in particular for lifesaving interventions. [11, 21, 22] Efforts should be made to increase knowledge and skills of staff at referral facilities on identification and intervention of lifesaving interventions along with access to equipment and medications.

A study conducted in Finland by Raj et al. [7] found that delays to healthcare facilities were related to sustaining injury at a public place. Similar results are illustrated in our study, although again, the results did not reach statistical significance. This could be explained by the fact that injuries at work or home will be transferred earlier to the initial hospital, and transfer to a trauma center will also be easier due to the presence and assistance of relatives/colleagues.

Several studies have confirmed that high ISS is related to poor outcomes [14–16]. As a result, these patients require prompt and early transfer. In our study, a slightly higher proportion of patients who had high ISS arrived within 6 hours as opposed to those with lower ISS, which is similar to Harrington's findings [6]. Limited management capacities at the peripheral facilities in terms of investigations and specialty services may explain the promptness of transfers [4].

The instability of the transferred patients on arrival was proved by the significant number of interventions needed to be carried out soon after arrival at EMD-MNH. This may be a surrogate marker of the inadequate care at the initial health facilities. Better infrastructure and availability of equipment in peripheral hospitals may help improve the care of polytrauma patients [3]. Moreover, efforts should be targeted at improving capacity to care for these polytrauma patients at lower-level health facilities, especially for initial stabilization.

A higher proportion of patients who came late (more than 6 hours) were injured during the day than at night. This is in contrast with studies conducted in HICs which show that the majority were injured during the night [19]. Our initial hypothesis was that injuries sustained at night would be more likely to be delayed in reaching the referral hospital because EMDs are generally less staffed at night and may have difficulty arranging transport or communicating with the referral center. These findings of greater delay during the day could be due to heavy traffic jams during the day in the commercial city of Dar es Salaam. Furthermore, a shortage of staffing during the night at peripheral facilities may precipitate earlier attempts to transfer to well-staffed facilities [4].

GCS less than 8 was associated with a sixteen-fold higher risk of mortality. In several studies conducted in both developed and developing countries, a low GCS has been found to be a predictor of mortality [11–13]. Moreover, patients with hypotension denoted by a SBP ≤90 mmHg had a seven times increased risk of mortality in our study. Similar findings were again noted in HICs and LMICs [11, 17]. These findings help to outline the role of vital signs in risk stratification of multiple trauma patients and their role to direct health professionals in the need for early identification, aggressive resuscitation measures, and early transfer to definitive care.

In our study, we found an overall 7-day mortality of twenty percent, which matched closely with the study carried out on polytrauma patients in Athens by Markopoulou et al. [17]. Lower mortality rates have also been noted in other studies of LMICs [2, 20]. The differences can be due to the fact that these studies included less severely injured patients, but our study only recruited polytrauma patients at national referral level health facilities.

From our study, timeliness did not seem to affect the outcome. Several reasons that could have contributed to this finding: First, patients with more severe injuries could have died either on scene, whilst at the initial facility or en-route to our facility and thus may not have been captured. Second, other factors such as GCS, hypotension, and hypoxia by themselves are strong predictors of death, and as such, a few hours' difference in the arrival of these patients may not affect their outcome. Another possibility could be that perhaps the original 6 hours cut off chosen may be too long as patients with life-threatening injuries could have died in the first few hours. Nevertheless, using time as a continuous variable, there was still no difference in the arrival of patients that survived and died.

## 5. Limitations

Being a single center study may affect generalizability. However, MNH is the main center for receiving severely injured polytrauma patients, and thus our study might cast a picture of the general presentations. Recall bias also could distort our results since referral forms did not always document the timings of injury, arrival, or transfer, and thus, these were sought from the patient/next of kin, or health professional accompanying the patient and thus subject to variation. The exclusion of nonreferral patients could also affect the observed results.

## 6. Conclusion

The majority of polytrauma patients arrive at the tertiary facilities delayed for more than 6 hours, and a distance of more than 8 km between facilities is associated with delay. Hypotension, hypoxia, and GCS of less than 8 are independent predictors of mortality. Despite of the delay, many polytrauma patients did not have the needed stabilization. Therefore, there is a need to expedite transfer of polytrauma patients to a center capable of providing care, and efforts should be made to improve pre-referral care provided at initial health facilities.

## Figures and Tables

**Figure 1:** Flowchart of the trauma patient who presented at EMD, MNH, Dar es Salaam, Tanzania.

**Table 1:** Demographic and clinical characteristics of referral polytrauma patients who presented to the EMD-MNH.

Variables	Frequency, *n* (%) *N* = 120
*Sex*	
Male	103 (85.8)

*Age groups*	
Median age (IQR)	30 (25–39)
18 to 33 years	72 (60.0)
34 to 49 years	35 (29.2)
More than 50 years	13 (10.8)

*Time of injury*	
Night^*∗∗*^	65 (54.2)

*Mechanism of injury*	
Motor vehicle accident	101 (84.2)
Motorcycle driver/passenger	59 (49.2)
Pedestrian	31 (25.8)
Car/truck/bus driver/passenger	11 (9.2)
Assault	11 (9.2)
Others (fall/GSW)	8 (6.6)

*Pattern of injury*	
Head/neck	107 (89.2)
Long bones/pelvis	82 (68.3)
Abdomen	28 (23.3)
Face	26 (21.7)

*Injury severity score*	
Median score (IQR)	29 (24–34)
Critical (≥25)	82 (68.3)
Severe (16–24)	38 (31.7)

*Glasgow Coma Scale*	
3 to 8	39 (32.5)
9 to 13	33 (27.5)
14 to 15	48 (40.0)

*Primary survey*	
Compromised airway	41 (34.2)
Compromised breathing	58 (48.3)
Compromised circulation	37 (30.8)
Compromised disability	88 (73.3)
Compromised exposure	86 (71.7)

Needed critical intervention within 15 mins of arrival	68 (56.7)

*Prereferral stabilization indicated but not performed*	
Cervical spine immobilization	54/88 (61.4)
Endotracheal intubation	38/41 (92.7)
Chest tube	17/17 (100.0)
Blood transfusion	28/32 (88.9)
Splinting	24/72 (33.3)
Intravenous fluids	22/120 (18.3)
Pelvic binder	12/12 (100.0)

**Table 2:** Referral characteristics and timing of presentation of referral polytrauma patients who presented to the EMD-MNH, Dar es Salaam, Tanzania.

Variables	Median (IQR)	Frequency, *n* (%) *N* = 120
*Distance between facilities*	8.1 (6.9–23.15)	
0 to 20 km		82 (68.3)
21 to 40 km		22 (18.3)
More than 40 km		16 (13.4)

*Time from injury to first hospital*		
Median time (minutes) (IQR)	40 (33–50)	
<60 mins		96 (80.0)
60–120 mins		24 (20.0)

*Length of stay at referring hospital*		
Median time (minutes) (IQR)	283 (240–350)	

*Overall time from injury to MNH*		
Median time (minutes) (IQR)	377 (314–469)	
≤360 minutes		55 (45.8)
>360 minutes		65 (54.2)

**Table 3:** Factors associated with timely presentation of referral polytrauma patients who presented to the EMD-MNH, Dar es Salaam, Tanzania.

Variables	Timely (*N* = 55)	Delayed (*N* = 65)	RR (95% CI)
*Age groups*			
18–33 years	32 (44.4)	40 (55.6)	0.9 (0.6–1.4)
>33 years	23 (47.9)	25 (52.1)	

Glasgow Coma Scale ≤8	18 (46.2)	21 (53.8)	1.0 (0.7–1.5)

Time of injury night	33 (50.8)	32 (49.2)	1.3 (0.8–1.9)

Needed intervention at EMD	34 (50.0)	34 (50.0)	1.2 (0.8–1.9)

*ISS*			
Critical (≥25)	39 (47.6)	43 (52.4)	1.1 (0.7–1.7)
Severe (16–24)	16 (42.1)	22 (57.9)	

*Location of injury*			
Public place	50 (43.9)	64 (56.1)	0.5 (0.3–0.8)
Work	5 (83.3)	1 (16.7)	

*Distance between facilities*			
<8 km	36 (54.5)	30 (45.5)	1.6 (1.1–2.4)
≥8 km	19 (35.2)	35 (64.8)	

*Level of referring facility*			
Regional hospital	17 (36.2)	30 (63.8)	2.0 (0.9–4.3)
District hospital	34 (53.1)	30 (46.9)	
Level II private	4 (44.4)	5 (55.6)	

**Table 4:** Univariate and multivariate analyses of predictors of mortality of referral polytrauma patients who presented to EMD-MNH.

Variable	Univariate, OR (95% CI), *P* value	Multivariate, AOR (95% CI), *P* value
Age >33 years	1.1 (0.4–2.7), 0.852	
Male sex	1.2 (0.3–4.5), 0.794	
GCS ≤8	**30.3 (8.2–112.8), <0.0001**	**16.3 (3.1–86.3), 0.001**
SpO2 ≤92%	**29.6 (6.5–134.9), <0.0001**	**8.3 (1.4–50.9), 0.022**
Heart rate ≤60 or ≥100	7.9 (1.7–35.3), 0.007	2.6 (0.4–19.4), 0.342
Respiratory rate ≤10 or >20	3.6 (1.3–10.6), 0.017	1.3 (0.3–6.0), 0.750
Systolic BP ≤90 mmHg	**8.3 (3.0–22.6), <0.0001**	**7.3 (1.6–33.6), 0.011**
Injury severity score (≥25)	5.8 (4.5–7.2), 0.998	
Needed intervention at EMD	7.3 (2.0–26.1), 0.002	0.7 (0.1–5.4), 0.763
Delayed >6 hrs	1.0 (0.4–2.5), 1.000	1.4 (0.3–5.6), 0.659

## Data Availability

The dataset supporting the results of this article is available from the authors on request.

## Abbreviations

CI: Confidence interval
EMD: Emergency medicine department
EMS: Emergency medical services
ESI: Emergency severity index
GCS: Glasgow Coma Scale
HICs: High income countries
IQR: Interquartile range
ISS: Injury severity score
Km: Kilometers
LMIC: Low- and middle-income countries
LOS: Length of stay
MNH: Muhimbili National Hospital
MOI: Muhimbili Orthopedic Institute
MUHAS: Muhimbili University of Health and Allied Sciences
OR: Odds ratio
RR: Relative risk
SBP: Systolic blood pressure
SpO2: Saturation
TC: Trauma center
UK: United Kingdom
USA: United States of America
WHO: World Health Organization.
